# Prevalence of *Pseudomonas aeruginosa* in Post-operative Wound Infection in a Referral Hospital in Haryana, India

This article has been retracted.

**DOI:** 10.4103/0974-2727.72153

**Published:** 2010

**Authors:** K Prabhat Ranjan, Neelima Ranjan, Satish K Bansal, D R Arora

**Affiliations:** Department of Microbiology, Maharaja Agrasen Medical College and Hospital, Agroha (Hisar),Haryana, India; 1 Department of Surgery, Maharaja Agrasen Medical College and Hospital, Agroha (Hisar),Haryana, India

**Keywords:** *Pseudomonas aeruginosa*, postoperative wound, prevalence, nosocomial, antibiotic

## Abstract

**Background:**

The objective of our study was to determine the prevalence of *Pseudomonas aeruginosa* in the isolates of postoperative wound and its susceptibility pattern to commonly used antibiotics.

**Materials and Methods:**

During a 2-year period, specimens were received as postoperative wound swabs in Microbiology Laboratory, Maharaja Agrasen Medical College, Agroha (Hisar), Haryana, India.

**Result:**

Of the 300 bacterial isolates, 89 (29.6%) were *P. aeruginosa*, followed by *Escherichia coli* (61, 20.3%), *Klebsiella* spp. (50, 16.6%), *Staphylococcus aureus* (43, 14.3%), *Proteus* spp. (19, 6.3%), *Acinetobacter* spp. (9, 3.0%), and *Citrobacter freundii* (2, 0.6%). There was no growth in 27 (9.0%) specimens.

**Conclusion:**

*P. aeruginosa* isolation was higher in male patients and most common in the age group of 21-40 years. The susceptibility pattern showed the organism to be most commonly susceptible to imipenem, followed by meropenem, cefoperazone/sulbactam, ticarcillin/clavulanate, and amikacin.

## INTRODUCTION

Postoperative wound infection or surgical site infection is an important cause of health care associated infections among surgical patients. Patients who develop wound infections have longer hospital stays, more expensive hospitalizations, and increased mortality.[1] The development of wound infections depends on the integrity and protective functions of the skin.[2]

*Pseudomonas aeruginosa* is a leading cause of health care associated infections, ranking second among gram-negative pathogens as reported by the United States national nosocomial infection surveillance system. *P. aeruginosa* contributes substantially to wound-related morbidity and mortality worldwide. The organism enters into the blood, causing sepsis that may spread to the skin and leads to ecthyma gangrenosum, a black necrotic lesion.[3] It produces several substances that are thought to enhance the colonization and infection of host tissue.[4] These substances together with a variety of virulence factors, including lipopolysaccharides (LPSs), exotoxin A, leukocidin, extracellular slime, proteases, phospholipase, and several other enzymes, make *P. aeruginosa* the most clinically significant pathogen among non-fermenting bacteria. *P. aeruginosa* has the capacity to carry plasmids containing genes that regulate antimicrobial resistance, and this feature has led to the appearance of some strains that are resistant to normally reliable antibiotics.[5] Out of these, there are multiple reasons for postoperative wound infections, which have been validated and documented as risk factors.

A risk factor is any recognized contribution to an increase in postoperative wound infection.[6] The virulence and invasive capability of the organisms have been reported to influence the risk of infection, but the physiological state of the tissue in the wound and immunological integrity of the host seem to be of equal importance in determining whether infection occurs or not.[7] Primary infections are usually more serious, appearing within 5–7 days of surgery. These infections are mostly related to endogenous flora and some other environmental sources in the operating theater. The deep-seated sepsis developing within 30 days after a surgery and before the wound has been dressed reflect a theater infection.[8] Some of the studies support the concept that a reduction in postoperative wound infection is directly related to increased education and awareness of its causes, and its prevention is greatly aided by critically evaluated infection control practice.[9]

The prevalence of primary wound infection is correlated to the bacteriological cleanliness of the operation. Clean operation (<2%) does not involve opening a viscous or cutting across mucus membranes. In contaminated operations (20%), a viscous normally containing bacteria or a membrane normally colonized with bacteria is incised, while in clean–contaminated operations (<10%), a viscous or membrane which is usually sterile, is incised.[10] Health care associated infections tend to be more superficial and frequently follow the dressing of wounds in the ward. Similarly, skin infections such as boils or abscesses developing at sites other than the operation site indicate that the infection was acquired in the ward.[7] Wound infection after contaminated operations is usually caused by the bacteria normally residing in the opened viscous or on the incised mucus membrane, i.e. the bacteria belong to the patient’s own normal flora, or have gained entry while the patient is in a hospital.[11] These include operations which are carried out through a field already contaminated by bacteria such as abscesses and colon operations.[10] Bacteriological studies have shown that postoperative wound infection is universal and that the bacterial types present vary with geographic location, bacteria residing on the skin, clothing at the site of wound, time between wound and examination.[12] Facultative anaerobic gram-negative bacilli, Streptococci and Staphylococci remain in the colon, regardless of the type of preparation. The bowel and postoperative infection in colon and rectal surgery without systemic intraoperative prophylaxis can be as high as 50%.

In the recent years, the growing incidence of *P. aeruginosa* has been of particular interest. The incidence of *P. aeruginosa* in postoperative wound infection is becoming more serious in developing countries because of lack of general hygienic measures, mass production of low quality antiseptic and medicinal solutions for treatment, and difficulties in proper definition of the responsibilities among the hospital staff.[13] The hospital-acquired nature of infections with *P. aeruginosa* has been noted and while some patients suffer endogenous infections, the vast majority is acquired from exogenous sources. So, the objective of our study was to determine the prevalence of *P. aeruginosa* in the isolates of postoperative wounds in our hospital and its antimicrobial susceptibility pattern.

## MATERIALS AND METHODS

The study was conducted in the bacteriology laboratory, Department of Microbiology, Maharaja Agrasen Medical College and Hospital, Agroha (Hisar), India. All the specimens received from patients hospitalized from April 2007 to March 2009 were processed for isolation and identification of bacterial pathogens, according to the standard microbiological techniques.[14]

### Clinical specimens

Postoperative wound swabs were collected aseptically with two sterile cotton wool swabs for each sample from different wards in the hospital. One swab was for Gram stain and the other one was for culture.

### Culture media and biochemical tests

The following media were used and tests were conducted in this study: blood agar, MacConkey agar, chocolate agar, nutrient agar, mannitol salt agar, Simmon citrate agar, peptone water, indole production test, motility test, methyl red test, voges proskauer test, catalase, coagulase, urease, and oxidase tests. All the above media and reagents were obtained from HiMedia, Mumbai, India. The media were prepared according to the manufacturers’ instructions.

All wound swabs collected for bacteriology investigations during the study period were treated according to the established methods of treating wound swabs. Gram stain preparations were made from one swab and culture are processed from another swab.

The plates were incubated at 37°C for 18–24 hours in an incubator. The plates were read the following day but extended to 48 hours if there was no bacterial growth within 24 hours. Isolated colonies were subjected to Gram staining and biochemical tests for identification.

Identification was carried out according to the standard biochemical tests.[14]

### Antibiotic susceptibility testing

Antimicrobial susceptibility test were carried out on isolated and identified colonies of *P. aeruginosa* using commercially prepared antibiotic disk (HiMedia) on Mueller Hinton agar plates by the disk diffusion method, according to the Central Laboratory Standards Institute (CLSI) guidelines.[15] Antibiotic testing was not done of other bacterial isolates in this study since our focus was on the prevalence of *P. aeruginosa*. The standard strain of *P. aeruginosa* (ATCC 27853) was used as a control. Antibiotics used in our study were piperacillin (100 µg), ceftazidime (30 µg), cefepime (30 µg), imipenem (10 µg), meropenem (10 µg), ampicillin/sulbactam (10/10 µg), piperacillin/tazobactam (100/10 µg), ticarcillin/clavulanate (75/10 µg), cefoperazone/sulbactam (75/10 µg), gentamicin (10µg), tobramicin (10 µg), amikacin (30 µg), and ciprofloxacin (5 µg).

## RESULTS

A total of 300 specimens were obtained from postoperative wounds, including superficial and deep-seated infections of all patients hospitalized at surgical, pediatrics, orthopedic, obstetrics, and gynecology wards.

### Isolation

The most common isolated organism from postoperative wounds was *P. aeruginosa* (89 isolates, 29.6%), followed by *Escherichia coli* (61 isolates, 20.3%), *Klebsiella* spp. (50 isolates, 16.6%), *Staphylococcus aureus* (43 isolates, 14.3%), *Proteus* spp. (19 isolates, 6.3%), *Acinetobacter* spp. (9 isolates, 3.0%), and *Citrobacter freundii* (2 isolates, 0.6%). There was no growth in 27 (9.0%) samples. The abscess drainage was the most common type of postoperative wound (17.90%), followed by the surgery of diabetic foot (12.82%), cesarean section (11.72%), and open knee surgical wound (11.35%) [Table 1].

**Table 1:** The number of wound swabs in relation to the type of surgery

Type of surgery	Number of specimens	Percentage
Abscess drainage	49	17.90
Diabetic foot	35	12.82
Cesarean section	32	11.72
Open knee wound	31	11.35
Liver abscess	23	8.42
Herniorrhaphy	17	6.22
Abdominal abscess	16	5.80
Nail removal	12	4.39
Perianal fistu	11	4.02
Septoplasty	10	3.66
Mastoidectomy	10	3.66
Neck abscess	7	2.56
Skin grafting	6	2.19
Lipoma excision	5	1.83
Bone excision	5	1.83
Thyroidectomy	4	1.46

The frequency of *P. aeruginosa* isolation in relation to age is shown in Table 2. The most frequent isolation of the *P. aeruginosa* was noted in the age group of 21–40 years (48.6%), followed by those in the age group of 41–60 years (40.6%), 0–20 years (5.0%), and >60 years (4.0%). We found the relationship between postoperative wound infections and sex. The prevalence rate was higher in male (58%) patients compared with females (42%).

**Table 2:** The frequency of *P. aeruginosa* isolation in relation to the age group

Age group (years)	Number of specimens	Number of isolation	Percentage
0–20	15	8	5.0
21–40	146	53	48.6
41–60	122	44	40.6
>60	17	7	4.0

### Susceptibility

*P. aeruginosa* was most commonly susceptible to imipenem (76.9%), followed by meropenem (70.4%), cefoperazone/sulbactam (62.1%), ticarcillin/clavulanate (60.7%), and amikacin (53%) [Table 3].

**Table 3:** The susceptibility pattern of *P. aeruginosa* isolated in postoperative wounds

Antibacterial	Percentage of susceptibility
Imipenem	76.9
Meropenem	70.4
Cefoperazone/sullbactam	62.1
Ticarcillin/clavulanate	60.7
Amikacin	53
Piperacillin/tazobactam	45.8
Ciprofloxacin	36
Ceftazidime	35.8
Tobramicin	30.5
Gentamicin	29.1
Cefepime	25.2
Piperacillin	13.6
Ampicillin/sulbactam	12

## DISCUSSION

A surgical wound infection is a postoperative complication that brings about embarrassment to the surgeon, considerable financial burden, undue discomfort to the patient, and sometimes death. Our study shows that *P. aeruginosa* was most prevalent (29.6%) among all the pathogens isolated from the surgical wound. Our results were consistent with similar studies carried out by Anupurba and colleagues which showed *P. aeruginosa* was isolated in 32% of isolates.[16] Oguntibegri and Nwobu, in their study, concluded it to be 33.3%[17] and Hani and colleagues found a prevalence rate of 27.78%.[18] Stephen and colleagues, in a similar study, reported a frequency of *P. aeruginosa* isolation rate of 18.8%.[19] We therefore report it as a significant finding which is in agreement with that obtained in other hospitals. The frequency of *P. aeruginosa* isolation was found to be maximal in patients who underwent cesarean section in the study by Oguntibeju and Nwobu[19] and in those with surgical wound infections and undergoing cesarean section in the study by Hani and colleagues.[20] In our study, it was most commonly isolated in procedures involving drainage of abscesses and diabetic foot operations, followed by cesarean section operations.

When factors such as age and sex of the patient were considered, we found the occurrence of *P. aeruginosa* to be higher in males and in patients in the age group 21–40 years. Stephen and colleagues found that *P. aeruginosa* was more commonly isolated from patients in the age group 21–30 years.[21] We found the prevalence rate to be higher in male (58%) patients compared to females (42%). Jamshaid and colleagues also reported that *P. aeruginosa* infections were more common in males, and Stephen and colleagues also reported in their study that male patients had higher isolation rates.[21]

The maximal susceptibility of *P. aeruginosa* isolates was against imipenem (76.9%) and meropenem (70.4%). Navaneeth and colleagues, in their study, noted 88% susceptibility against each of imipenem and meropenem, among *P. aeruginosa* isolates.[22] Bonfiglio and colleagues, in their study, summarized that meropenem was the most active compound against *P. aeruginosa* isolates, followed by amikacin.[23] Although we found carbapenems to be the most successful drugs in vitro against *P. aeruginosa*, there is a likelihood of resistance to even these as seen in studies carried out on multidrug-resistant phenotype of *P. aeruginosa*.[24] Resistance to carbapenems is most likely to occur by the interplay of excess β-lactamase production, impermeability via a loss of porin protein Opr D, together with the up-regulation of multidrug efflux systems, primarily MexA MexB Opr M.[25] Our study shows that there is an increased rate of incidence of *P. aeruginosa* in postoperative wound infections. The most common causative agent of postoperative infections was *P. aeruginosa*, followed by *E. coli*, *Klebsiella* spp., *S. aureus*, *Proteus* spp., and *Acinetobacter* calcoaceticus. Other less common causes were *Streptococcus pyogenes, Enterococcus faecalis* and *C. freundii*^26^. This is in agreement with survey studies carried out in various hospitals. The infection appears to be common in hospitals with relaxed hygienic measures and is dependent on age, sex and even duration of stay in the hospital. The primary reason for this increase in postoperative infection rate with prolonged preoperative hospitalization may be the colonization of patients with hospital-acquired resistant microorganisms.
